The article "Effect of CLIC1 gene silencing on proliferation, migration, invasion and apoptosis of human gallbladder cancer cells" was retracted in 2021. Reasons: duplicated images; unreliable results or conclusions; concerns about the data.

# Effect of CLIC1 gene silencing on proliferation, migration, invasion and apoptosis of human gallbladder cancer cells

**DOI:** 10.1111/jcmm.13499

**Published:** 2018-03-08

**Authors:** Yue‐Ming He, Zhong‐Lin Zhang, Quan‐Yan Liu, Yu‐Sha Xiao, Lei Wei, Chen Xi, Xiang Nan

**Affiliations:** ^1^ Department of Hepato‐Pancreato‐Biliary Surgery Zhongnan Hospital of Wuhan University Wuhan China; ^2^ College of Life Science Wuhan University Wuhan China

**Keywords:** CLIC1 gene silencing, gallbladder cancer, GBC‐SD cell, apoptosis, proliferation, migration, invasion

## Abstract

This study aimed to explore the effects of CLIC1 gene silencing on proliferation, migration, invasion and apoptosis of human gallbladder cancer (GBC). GBC and normal gallbladder tissues were extracted for the detection of mRNA and protein expressions of CLIC1. GBC‐SD and NOZ cells in the logarithmic growth phase were selected to conduct the experiment. Three different siRNA recombined expression vectors were established using CLIC1 as a target at different sites. Reverse transcription quantitative polymerase chain reaction (RT‐qPCR) and Western blotting were, respectively, used to detect the CLIC1 mRNA and protein expressions. MTT assay was performed to detect the cell proliferation. Flow cytometry was applied to measure the cell apoptosis and cell cycle distribution. The variations of cell migration and invasion were evaluated using Transwell assay. GBC tissues showed higher CLIC1 mRNA and protein expressions than normal gallbladder tissues. The CLIC1 mRNA and protein expressions in the CLIC1 siRNA group were significantly lower than those in the NC and blank groups. Compared with the NC and blank groups, the CLIC1 siRNA group showed a significant decrease in cell proliferation but an obvious increase in apoptosis rate in GBC cells. Besides, in the CLIC1 siRNA group, cell percentage in G0/G1 and G2/M phase was gradually increased but decreased in S phases. The migration and invasion abilities in GBC cells were significantly lower than those in the NC and blank groups. Our study demonstrates that CLIC1 gene silencing could promote apoptosis and inhibit proliferation migration and invasion of GBC cells.

## Introduction

GBC, a type of malignant tumour with weak prognosis, is reported to rank the seventh most common carcinoma all over the world 1, 2. There are some relative symptoms that may be the marker of malignant GBC, including jaundice and a pain in the abdomen as well as sometimes an obvious abdominal mass that appears at a late stage of this disease 3. At present, many treatment methods have been investigated on the treatment of GBC 4, 5. It has been reported that palliative operation, endoscopic as well as radiologic bypass methods were used for patients with unresectable GBC, and the combined radiation and chemotherapy and systemic chemotherapy are also adopted as managements for advanced tumours 6. How to effectively inhibit proliferation and induce apoptosis of GBC cells is always the focus of the researchers for exploring the treatment of GBC, including using Lupeol under the suppression of EGFR/MMP‐9 signalling pathway as well as applying a demethylated form of cantharidin called norcantharidin 7, 8.

The article "Effect of CLIC1 gene silencing on proliferation, migration, invasion and apoptosis of human gallbladder cancer cells" was retracted in 2021. Reasons: duplicated images; unreliable results or conclusions; concerns about the data.

There we also tried to find a potential alternative to promote apoptosis and inhibit proliferation of GBC cells. Actually, chloride intracellular channel 1 (CLIC1), a metamorphic protein acting as cell oxidation sensor and playing an important role in inflammation, has been reported to be capable of participating in the progress of cell division and motility and it is likely that this gene is involved in modulating tumorigenesis 9, 10. In addition, this newly discovered member of the chloride channel protein family has been implicated in multiple human cancers such as pancreatic cancer, gastric cancer as well as hepatocarcinoma, and in colon cancer, it was also unfolded to be responsible for regulating the migration and invasion of the cancer cells 11, 12, 13, 14. Some researchers have found that CLIC1 could function as a biomarker for some cancers such as epithelial ovarian cancer 15. Therefore, considering the properties of CLIC1 gene in cell modulation and its involvement in tumorigenesis, we have been suggested that in GBC, CLIC1 gene silencing may have some effects on the biological behaviours of GBC cells. This study is designed to evaluate whether the use of CLIC1 gene silencing could produce an inducing effect on apoptosis and an inhibitory one on proliferation of GBC cells, which may provide a new light on gene therapy in the treatment of GBC.

## Materials and methods

### Ethics statement

This study was approved by the Clinical Experiment Ethics Committee of Zhongnan Hospital of Wuhan University, and all the participants provided informed consent before participating in the study.

### Sample preparation

Eighteen normal gallbladder tissues were harvested from patients with benign diseases, and 28 GBC tissues were collected from patients with GBC. All of these surgically resected tissues were from Zhongnan Hospital of Wuhan University. After washed with normal saline, all extracted tissues were cut into 1.0 × 1.0 × 1.0 cm pieces and stored in liquid nitrogen. The study was approved by the Institutional Review Board of our hospital.

### Cell culture, screening and grouping

GBC‐SD, EH‐GB1, NOZ and SGC‐996 cells were purchased from American Type Culture Collection (ATCC) and diluted by 10 times using RPMI 1640 culture solution (Thermo Fisher Scientific, Beijing, China). Cell suspension was realized by blowing and beating. The cells received a low‐speed centrifugation (1000 rpm) for 8 min. (Heeaeus Company, Hanau, Germany), which was repeated thrice, and then the sediment cells were transferred into the culture bottle (Thermo Fisher Scientific, Beijing, China), adhering to the wall in Dulbecco's minimum essential medium (DMEM) sugar culture solution (31600‐034, Hyclone, Logan city, Utah, USA) with 10% heat‐inactivated foetal bovine serum (FBS) and 100 U/ml penicillin and 100 μg/ml streptomycin. They were cultured in an incubator (SHEL LAB, Portland, Oregon, USA) with the temperature of 37°C and saturated humidity of 5% CO_2_. RT‐qPCR was employed to detect how CLIC1 expressed in the four cell lines including GBC‐SD, EH‐GB1, NOZ and SGC‐996. The two cell lines in which CLIC1 expressed the highest were selected for further experiment. Every 2–3 days, GBC cells that were transfected with control siRNA were established as the negative control (NC) group, and GBC cells that did not transfect any plasmids were selected as the blank group. The cells were cultured in an incubator for 48 hrs. After the CLIC1 siRNA group (GBC‐SD cells transfected with CLIC1 siRNA) was cultured for 10–12 hrs, the culture medium containing siRNA‐Lipofectamine 2000 mixture was replaced with the fresh one.

The article "Effect of CLIC1 gene silencing on proliferation, migration, invasion and apoptosis of human gallbladder cancer cells" was retracted in 2021. Reasons: duplicated images; unreliable results or conclusions; concerns about the data.

### Observation of cell number and morphology under an inverted microscope

Cells in logarithmic growth phase were selected and incubated in the 24‐well culture plate. When the cells were adherent to the wall, the morphology of GBC cells in the NC and CLIC1 siRNA groups was observed using the inverted microscopes (Olympus Co., Ltd., Beijing, China).

### Model establishment of CLIC1 siRNA

GBC cells, which were possessed with CLIC1 expression, were selected. The siRNA Designer System from Shanghai Genepharma, Co., Ltd, Shanghai, China, was applied to make the preliminary selection of siRNA sequences based on CLIC1 (NM_001288.4) gene information. Rational design principle proposed by Reynolds was used for manual selection among the preliminarily selected sequences. Finally, four sequences were chosen for this experiment. Meanwhile, the base sequence of the selected siRNA was rearranged to make sure that there was no homology‐based method between the selected one and the other genes for designing a NC. The designed siRNA was sent to Shanghai Genepharma, Co., Ltd (Table 1), and manipulated using Lipofectamine 2000 (Invitrogen Inc., Carlsbad, CA, USA). According to the instructions, siRNA‐Lipofectamine 2000 was used for transfecting GBC cells.

The article "Effect of CLIC1 gene silencing on proliferation, migration, invasion and apoptosis of human gallbladder cancer cells" was retracted in 2021. Reasons: duplicated images; unreliable results or conclusions; concerns about the data.

**Table 1:** Information for siRNA sequences

Sequence tags	Sequences (5′‐3′)	
CLIC1 siRNA 1	Sense	GAGCUUGUGUUGUGCUGAATT
	Antisense	UUCAGCACAACACAAGCUCTT
CLIC1 siRNA 2	Sense	CAGCACUCAAUGACAAUCUTT
	Antisense	AGAUUGUCACUCAAUGCUGTT
CLIC1 siRNA 3	Sense	GCCAAAGUUACACAUAGUATT
	Antisense	UACUAUGUGUAACUUUGGCTT
CLIC1 siRNA 4	Sense	GGACAACAUAUUUCAGUAATT
	Antisense	UUACUGAAAUAUGUUGUCCTT
CLIC1 siRNA NC	Sense	UUCUCCGAACGUGUCACGUTT
	Antisense	ACGUGACACGUUCGGAGAATT

NC, negative control; CLIC1, chloride intracellular channel 1.

### Transfection efficiency observed by a fluorescent inverted phase contrast microscope

The well‐grown GBC cells in the CLIC1 siRNA group and the NC group were selected. After the old culture medium was removed, the phosphate buffer saline (PBS) (Beyotime Institute of Biotechnology Co., Ltd., Shanghai, China) was used for rinsing the cells for two to three times, and the new DMEM culture medium containing 10% FBS without antibiotics was added. Fluorescence in each well was observed by a fluorescent inverted phase contrast microscopy, and the pictures were taken as well. The percentage of fluorescent cells in the total cells (transfection efficiency) was calculated.

### RT‐qPCR

Tissues and GBC cells of the third generation that grew well adhering to the wall were selected. Kits for RNA (GIBCO Company, NY, USA) were applied to extract RNA of the cells. RNA sediment was then dried in air for 5 min. and added with 25 μl double distilled water without RNA enzyme which dealt with diethyl pyrocarbonate (DEPC) (Sigma‐Aldrich Company, Louis, MO, USA). RNA was shaken for several times and dissolved. DNA/RNA tester (Beckman Coulter, Fullerton, CA, USA) was used to measure the absorbance value at the wavelength of 260 nm. RNA concentration was tested according to the formula. The response solutions were operated in the 2 ml centrifugation tube including 4 μl 5× reverse transcriptase buffer (Mg^2+^), 2 μl mixed solution of deoxynucleoside triphosphates (dNTP) (10 Mm for each), 1 μl Oligo dT Primer (10 pmol/l), 0.5 μl RNase inhibitor, 5 μl template RNA and ammonium metavanadate (AMV) reverse transcriptase. At last, DEPC water was added to reach a total volume of 20 μl and cDNA was synthesized. According to the bibliography, the primer of CXCR4 gene and the internal control β‐actin were synthesized by Shanghai Boya Biotechnology Co., Ltd. (Table 2). Response solution of 30 μl was prepared, including 0.15 μl Takara Taq HS (5 U/μl) (Takara, Japan), 3 μl 10× PCR buffer (Mg^2+^ Plus), 2.4 μl dNTP mixture (2.5 mM for each), 0.5 μl forward and reverse primers of the target gene for each (20 pM), 0.5 μl forward and reverse primers of β‐actin for each (20 pM), 3 μl template cDNA and 19.45 μl double distilled water. Pre‐denaturation was performed followed by denaturation, annealing and extension. After these responses, DNA ladder (molecular weight: Marker) and PBS solution, which used as NC, were added in the two sides of electrophoresis lane with a concentration of 1.2% agarose gel electrophoresis. Electrophoresis was performed at 80 mv and when it was finished, gel imaging system was applied to take pictures and analyse the density value of band. The expression of mRNA is equal to the density value of band in the target gene/density value of band in β‐actin.

The article "Effect of CLIC1 gene silencing on proliferation, migration, invasion and apoptosis of human gallbladder cancer cells" was retracted in 2021. Reasons: duplicated images; unreliable results or conclusions; concerns about the data.

**Table 2:** Primer sequences for RT‐qPCR

Genes	Sequences (5′‐3′)	Length of products
CLIC1	F: AATCAAACCCAGCACTCAATG	153 bp
	R: CAGCACTGGTTTCATCCACTT	
β‐actin	F: ACCAACTGGGACGACATGGAG	203 bp
	R: GTGAGGATCTTCATGAGGTAGTC	

F, forward; R, reverse; RT‐qPCR, reverse transcription quantitative polymerase chain reaction; CLIC1, chloride intracellular channel 1.

### Western blotting

CLIC1 expression in tissues and cells were detected using Western blotting. Culture bottles (BD Company, NY, USA) of 1 × 10^7^ GBC cells transfected by siRNA 3 with a 48‐hr response period were collected. The transfection solution without siRNA 3 was used as blank control. Protein extraction kit (Wuhan Boster Biological Technology Co., Ltd., Wuhan, China) was used for extracting proteins, and then, bicinchoninic acid (BCA) kit (Wuhan Boster Biological Technology Co., Ltd., Wuhan, Hubei, China) was applied to test protein content. The extracted proteins were separated by electrophoresis using 10% polyacrylamide gel (Wuhan Boster Biological Technology Co., Ltd., Wuhan, Hubei, China). After membrane transference was finished, they were placed on the horizontal table and immersed in sealing fluid for 1 hr (using a 5% concentration of bovine serum albumin diluted by PBS or evaporated skimmed milk as sealing fluid). The sealed polyvinylidene difluoride (PVDF) membrane was taken out and added with the primary antibody (AC106, Beyotime Institute of Biotechnology Co., Ltd., Shanghai, China) diluted with 5% bovine serum albumin at 100 μl/cm^2^ overnight at 4°C. The secondary antibody (A7007, Beyotime Institute of Biotechnology Co., Ltd., Shanghai, China) diluted with 5% bovine serum albumin at 100 μl/cm^2^ was added on the table and sealed for 1 hr at room temperature. The test kit A and B were mixed together at the proportion of 1: 1 in the culture dish, avoiding strong lights during the whole process. PVDF membrane immersed in PBS was placed in chemiluminescence (ECL) working solution for imaging. Bio‐Rad GelDoc 2000 Gel Imaging System was used to scan PVDF membrane (Bio‐Rad Laboratories, Hercules, CA, USA). After imaging, the Image Lab was used for image analysis and processing so as to quantitatively analyse the grey value of protein bands, with the grey value of β‐actin band as the control.

The article "Effect of CLIC1 gene silencing on proliferation, migration, invasion and apoptosis of human gallbladder cancer cells" was retracted in 2021. Reasons: duplicated images; unreliable results or conclusions; concerns about the data.

### 3‐(4,5‐dimethylthiazol‐2‐yl)‐2,5‐diphenyltetrazolium bromide (MTT) assay

Through experimental selection, siRNA 3, the best one to interfere CLIC1 gene, was used to transfect the GBC cells and digested with 0.25% pancreatin and diluted into single‐cell suspension with PBS. GBC cells were seeded in a 96‐well culture plate with a cell density of 2 × 10^4^ cells in each well (100 μl) and then cultured in an incubator at 37°C with saturated humidity of 5% CO_2_. After the cells were completely adhered to the wall, GBC cells in NC group were transfected 100 μl control siRNA and those in the CLIC1 siRNA group were transfected 100 μl CLIC1 siRNA. The blank group was conducted with no transfection but added with 100 μl RPMI 1640 culture solution. Each well was set with two wells and in every 96‐well plate, two wells were kept for receiving only 200 μl culture solution without adding cells, which was working as null‐balance. At 48 hrs after culture cells were transfected with siRNA 3, they were taken out of the plate. Each well in the 96‐well plate was added with 20 μl MTT solution (5 mg/ml) (AR1156, Wuhan Boster Biological Technology Co., Ltd.). After the cells were cultured for 4 hrs at 37°C, the culture solution in the well was poured out, and each well was added with 150 μl dimethyl sulfoxide (DMSO), allowing the plate to shake on the table for 8 min. After the crystal was fully dissolved, the blank wells were adjusted to zero. Enzyme‐linked immunosorbent assay (ELISA) was used to test the optical density (OD) value of each well and to analyse the cell inhibition rate and survival rate at the wavelength of 490 nm. Formula was as follows: proliferation rate is equal to the A value in the case group/the A value in the blank control group × 100%.

### Annexin V/propidium iodide (PI) staining

GBC cells transfected with siRNA 3 were seeded into a 12‐well plate at a cell density of 1 × 10^6^ per ml (BD Company, NY, USA). Each well was respectively added with 2 ml cell suspension and 2 ml siRNA 3 transfection working solution. After the cells were cultured for 48 hrs in the incubator, the cell suspension of 1 ml was centrifuged at 1000 rpm and 4°C for 10 min. Then the supernatant was abandoned and 1 ml cold PBS was added. Slow shaking was conducted to suspend the cells and then followed by the centrifugation at 1000 rpm and 4°C for 10 min. again and the supernatant was abandoned, which was repeated for two times. Cells were suspended using 200 μl PBS and added 10 μl Annexin V‐FITC (Beijing Biosea Biotechnology co., LTD., Beijing, China) and gently mixed up. This chemical response lasted for 15 min. at room temperature avoiding lights. PBS of 300 μl and 5 μl PI (Promega Company, Madison, Wisconsin, USA) was added, and flow cytometry was used to detect cell apoptosis.

The article "Effect of CLIC1 gene silencing on proliferation, migration, invasion and apoptosis of human gallbladder cancer cells" was retracted in 2021. Reasons: duplicated images; unreliable results or conclusions; concerns about the data.

### Flow cytometry

GBC cells transfected with siRNA 3 were seeded into a 24‐well plate at a cell density of 1 × 10^5^ per ml (BD Company, NY, USA). Each well was respectively added with 1 ml cell suspension. There were two groups with three wells in each group. After incubation for 48 hrs at 37°C and 5% CO_2_ saturated humidity, the cells were rinsed once with PBS which was then removed by centrifuging and were fixed at 4°C with 70% ethanol for 1 hr. The centrifugation was performed to remove the fixative and with PBS to rinse the cells for three times. PBS was removed by centrifuging and RNA enzyme was then added at 37°C, receiving water bath for 30 min. Afterwards, 800 μl PI was added and mixed up. The cells were restored at 4°C, being protected from light for 30 min. Flow cytometry was used to detect the cell cycle.

### Transwell assay

The cell density reached 3 × l0^5 ^cells/ml by cell suspension serum‐free culture medium. The cells were placed at the temperature of 37°C for 24 hrs and cultured in the incubator with 5% CO_2_. After that, the Transwell chamber was taken out. Ultraviolet lamp was used to light the front and back of the chamber for 3 hrs on the clean bench. Then, the chamber was placed in the corresponding well of the 24‐well plate. Each group was added with 100 pl cultured cells. The lower chamber was added with RPMI 1640 complete medium containing 10% FBS and 10 ttg/ml FN (Beijing Biosea Biotechnology Co., Ltd.) and they were placed in the incubator receiving culture for 24 hrs. Afterwards, the Transwell chamber was taken out. The remaining culture medium and the non‐transferred cells were removed. The selected cells were dried at room temperature for 30 min. and immersed in the 24‐well plate with 1% crystal violet solution, receiving a 20‐min. dye and PBS rinse. The microscope was used for counting the cells penetrating through the membrane in the Transwell chamber membrane, and the migration ability was detected under the microscope after extracellular matrix (ECM) gel was thawed at the last 4°C.

### Statistical analysis

SPSS 21.0 statistical software (IBM Corp. Armonk, NY, USA) was used for data analysis. Measurement data were presented as mean ± standard deviation (S.D.)The comparisons between two groups in measurement data with the normal distribution were analysed using *t‐*test. One‐way analysis of variance (ANOVA) was applied for the comparisons among multiple groups. The enumeration data were presented by percentage and analysed by chi‐square test. The significance level was set at *P *<* *0.05.

The article "Effect of CLIC1 gene silencing on proliferation, migration, invasion and apoptosis of human gallbladder cancer cells" was retracted in 2021. Reasons: duplicated images; unreliable results or conclusions; concerns about the data.

## Results

### CLIC1 expressed at a high level in DBC tissues

As presented in Figure 1, RT‐qPCR and Western blotting results revealed that, in comparison with normal gallbladder tissues, the mRNA and protein expressions of CLIC1 were dramatic up‐regulated in GBC tissues (*P *<* *0.05).

**Figure 1:** CLIC1 mRNA and protein expressions in GBC and normal gallbladder tissues. (**A**) RT‐qPCR of CLIC1 mRNA expression; (**B**) statistical results of CLIC1 protein expression; (**C**) Western blotting of CLIC1 protein expression; *compared with normal gallbladder tissues, *P *<* *0.05.

### CLIC1 expression in GBC‐SD, EH‐GB1, NOZ and SGC‐996 cell lines

The results of CLIC1 expression in GBC‐SD, EH‐GB1, NOZ and SGC‐996 cell lines are showen in Figure 2. CLIC1 expression in EH‐GB1 and SGC‐996 cell lines was significantly lower than that in GBC‐SD and NOZ. Therefore, GBC‐SD and NOZ cell lines were prepared for the following experiment.

**Figure 2:** CLIC1 expressions in GBC‐SD, EH‐GB1, NOZ and SGC‐996 cell lines. *compared with GBC‐SD and NOZ cell lines, *P *<* *0.05.

### mRNA expression of CLIC1 in GBC cells at different time‐points in each group

The results of RT‐qPCR showed that the CLIC1 mRNA expression in GBC‐SD and NOZ cells at 24, 48 and 72 hrs after transfection in the CLIC1 siRNA group was significantly lower than that in the NC and blank groups (all *P *<* *0.05). However, there was no significant difference between the NC and blank groups (*P *>* *0.05). Besides, the results were similar between GBC‐SD and NOZ cells (Fig. 3).

**Figure 3:** mRNA expression of CLIC1 at different time‐points in the CLIC1 siRNA, NC and blank groups. (**A**) CLIC1 mRNA expression in GBC‐SD cells at 24, 48 and 72 hrs after transfection; (**B**) CLIC1 mRNA expression in NOZ cells at 24, 48 and 72 hrs after transfection; *compared with the NC and blank groups, *P *<* *0.05.

### CLIC1 protein expression in GBC cells in the blank, NC and CLIC1 siRNA group

The results of Western blotting showed that the CLIC1 protein expression in GBC‐SD and NOZ cells at 24, 48 and 72 hrs after transfection in the CLIC1 siRNA group was significantly lower than that in the NC and blank groups (all *P *<* *0.05). However, there was no significant difference between the NC and blank groups (*P *>* *0.05). Besides, the detection results were same between GBC‐SD and NOZ cells (Fig. 4).

**Figure 4:** Protein expression of CLIC1 at different time‐points in the CLIC1 siRNA, NC and blank groups. (**A**) Western blotting of CLIC1 protein expression in GBC‐SD cells; (**B**) statistical results of CLIC1 protein expressions in GBC‐SD cells; (**C**) Western blotting of CLIC1 protein expression in NOZ cells; (**D**) statistical results of CLIC1 protein expressions in NOZ cells; *compared with the NC and blank groups, *P *<* *0.05.

The article "Effect of CLIC1 gene silencing on proliferation, migration, invasion and apoptosis of human gallbladder cancer cells" was retracted in 2021. Reasons: duplicated images; unreliable results or conclusions; concerns about the data.

### Transfection efficiency and growth state of GBC‐SD and NOZ cells in the CLIC1 siRNA, NC and blank groups

Lipofectamine 2000 transfected cells were selected and placed into the culture bottle in an incubator. After 48‐hr culture, the inverted microscope showed that there were a large number of cells in the CLIC1 siRNA, NC and blank groups. The nucleus was found comparatively large, and the cytoplasm was detected abundant in good growing state, which was able to participate in the following researches. The results of the fluorescent inverted phase contrast microscope showed that GBC‐SD and NOZ cells in the CLIC1 siRNA group were with slight fluorescence and diffused around the cells. The cells with fluorescence were also observed to be with coarse profile and some visible fluorescence inside the cells (Fig. 5). It proved that GBC‐SD and NOZ cells in the CLIC1 siRNA group were all successfully transfected with siRNA‐Lipofectamine 2000 with an average 48‐hr transfection rate at 80%.

**Figure 5:** Transfection efficiency and growth state of GBC‐SD and NOZ cells in the CLIC1 siRNA, NC and blank groups under a fluorescent inverted phase contrast microscope.

### CLIC1 siRNA inhibited proliferation of GBC‐SD and NOZ cells *in vitro*

The MTT assay results showed that the rate of GBC‐SD cell proliferation in the CLIC1 siRNA group at 24, 48 and 72 hrs after transfection was 14%, 29% and 39%, respectively. The rate of GBC‐SD cell proliferation in the NC group at 24, 48 and 72 hrs after transfection was 42%, 61% and 73%, respectively, and in the blank group, it was 43%, 56% and 69%, respectively. The rate of NOZ cell proliferation in the CLIC1 siRNA group at 24, 48 and 72 hrs after transfection was 12%, 26% and 35%, respectively. The rate of NOZ cell proliferation in the NC group at 24, 48 and 72 hrs after transfection was 40%, 60% and 70%, respectively, and in the blank group, it was 41%, 52% and 63%, respectively. Compared with the NC and blank groups, at each time‐point, the rate of cell proliferation was significantly lower in the CLIC1 siRNA group (all *P *<* *0.05, Fig. 6).

**Figure 6:** Cell proliferations in the CLIC1 siRNA, NC and blank groups by MTT assay. (**A**) cell proliferation rate in GBC‐SD cells; (**B**) cell proliferation rate in NOZ cells; *compared with the NC and blank groups, *P *<* *0.05.

The article "Effect of CLIC1 gene silencing on proliferation, migration, invasion and apoptosis of human gallbladder cancer cells" was retracted in 2021. Reasons: duplicated images; unreliable results or conclusions; concerns about the data.

### CLIC1 siRNA promoted apoptosis of GBC‐SD and NOZ cells

After 48‐hr transfection, the results of cell apoptosis in each group (Fig. 7) suggested that the apoptosis rate in the CLIC1 siRNA group was significantly higher than that in the NC and blank groups (both *P *<* *0.05). However, there was no significant difference between NC and blank groups in the cell apoptosis (*P *>* *0.05).

**Figure 7:** Cell apoptosis at 48^ ^hrs after transfection in the CLIC1 siRNA, NC and blank groups by flow cytometry. (**A**,** C**) cell apoptosis of GBC‐SD and NOZ in the CLIC1 siRNA, NC and blank groups by flow cytometry; (**B**,** D**) the bar chart of GBC‐SD and NOZ cells apoptosis rate in the CLIC1 siRNA, NC and blank groups; *compared with NC and blank groups, *P *<* *0.05.

### CLIC1 siRNA inhibited GBC‐SD and NOZ cell cycle

After 48‐hr transfection, the percentage of cell cycle distribution in the G2/M phase in the CLIC1 siRNA group amounted to 16.4 ± 1.6%. Compared with the NC and blank groups, the percentage of that in the G2/M phase was significantly increased in the CLIC1 siRNA group (both *P *<* *0.05). This revealed that the inhibition of the expression of CLIC1 gene could affect the progress of cell cycle to reduce the cells in S phase and to increase the cells in G0/G1 phase and G2/M phase (Fig. 8).

**Figure 8:** Cell cycle distributions at 48^ ^hrs after transfection in the CLIC1 siRNA, NC and blank groups by flow cytometry. (**A**,** C**) flow cytometry results of GBC‐SD and NOZ cell migration (200×); (**B**,** D**) statistical results of GBC‐SD and NOZ cell cycle; *compared with the NC and blank groups, *P *<* *0.05.

### CLIC1 siRNA inhibited the migration of GBC‐SD and NOZ cells

After 48‐hr transfection, the number of cells that had migrated through the Transwell chamber membrane in the CLIC1 siRNA group was decreased as compared with the NC and blank groups (*P *<* *0.05) (Fig. 9). The results revealed that CLIC1 gene silencing could impair the cell migration ability of GBC‐SD and NOZ cells.

**Figure 9:** Cell migrations at 48 hrs after transfection in the CLIC1 siRNA, NC and blank groups by Transwell assay. (**A**,** C**) results of GBC‐SD and NOZ cell migration under microscope (200**×**); (**B**,** D**) statistical results of GBC‐SD and NOZ cell migration; *compared with the NC and blank groups, *P *<* *0.05.

### CLIC1 siRNA inhibited the invasion of GBC‐SD and NOZ cells

After 48‐hr transfection, the number of cells that had invaded through the Transwell chamber membrane in the CLIC1 siRNA group was decreased as compared with the NC and blank groups (*P *<* *0.05) (Fig. 10). The results revealed that CLIC1 gene silencing could impair the cell invasion ability of GBC‐SD and NOZ cells.

The article "Effect of CLIC1 gene silencing on proliferation, migration, invasion and apoptosis of human gallbladder cancer cells" was retracted in 2021. Reasons: duplicated images; unreliable results or conclusions; concerns about the data.

**Figure 10:** Cell invasions at 48 hrs after transfection in the CLIC1 siRNA, NC and blank groups by Transwell assay. (**A**,** C**) results of GBC‐SD and NOZ cell invasion in three groups under a microscope (200×); (**B**,** D**) statistical results of GBC‐SD and NOZ cell invasion in three groups; *compared with the NC and blank groups, *P *<* *0.05.

## Discussion

GBC, in spite of its rarity in general, is regarded as a malignancy that is the most common of the biliary tract, which accounts for up to 80–95% of biliary tract cancers 16. According to the previous study, CLIC1 protein has been reported to be a sort of potential prognostic biomarker for hydatidiform moles that were transformed malignantly 17 **.** Therefore, it is likely to take silencing of CLIC1 into consideration for preventing and inhibiting the occurrence of GBC. In this study, we investigated the effects of CLIC1 gene silencing on the proliferation, migration, invasion and apoptosis of GBC cells *in vitro*.

The result showed that the mRNA and protein expressions of CLIC1 in the CLIC1 siRNA group were significantly lower than those in the NC and blank groups. There was another study which provided a consistent result, revealing that the CLIC1 siRNA was capable of suppressing the protein expressions and the CLIC1 mRNA at an effective rate 18. It was also reported that CLIC1 mRNA and protein expression were significantly decreased in the normoxia control group, suggesting a key role of CLIC1 silencing in colon cancer cells 19. One of the possible mechanisms might be that the CLIC1 protein expression was modulated by Cl (‐) current which could be prevented by the use of siRNA and thus resulted in a lower expression in the CLIC1 siRNA group compared with that in the NC and blank groups 10, 20.

In addition, compared with NC and blank groups, in the CLIC1 siRNA group, cell percentage in G0/G1 and G2/M phase was gradually increased but decreased in S phases. Besides, the CLIC1 siRNA group showed a significant decrease in GBC cell proliferation but an obvious increase in apoptosis rate. A similar research result could be found stating that CLICs, including CLIC1, which function as membrane regulated by actin, were possessed with an ability of modifying solute transport at crucial stages in the course of cellular events such as cell apoptosis, organelle and cell fusion and division, cell movement as well as cell‐volume modulation 21. It was also reported that CLIC1 could be a sort of soluble glutathione called S‐transferase‐like canonical fold 22. Actually, CLIC is able to shift into a transmembrane protein from a soluble cytoplasmic one, with its multimerises forming chloride ion channels that are selective when it is inserted into membranes 23. Thus, we speculated that it is by changing soluble cytoplasmic factors, regulating solute transport that CLIC1 is involved in the growth cycle of GBC cells, having something to do with the cell percentage at different phases. Consequently, the silencing of CLIC1 could produce an inhibitory effect on transporting GBC cell proliferation but a promoting impact on cell apoptosis.

The article "Effect of CLIC1 gene silencing on proliferation, migration, invasion and apoptosis of human gallbladder cancer cells" was retracted in 2021. Reasons: duplicated images; unreliable results or conclusions; concerns about the data.

Our results also demonstrated that CLIC1 gene silencing could impair the cell invasion ability of GBC cells. These results were in consistency with another one unfolding that silencing CLIC1 gene combined with shRNA could produce an effect on reducing cell migration and invasion and that one of the potential mechanisms through which CLIC1 gene expression regulates cell invasion was used to modulate the carcinoma suppressor maspin, annexin A7, matrix metalloproteinases as well as gelsolin 24 **.** What's more, CLIC1, as a member of CLIC family which is famous for its existence majorly as soluble proteins, has also been reported to be able to automatically insert into cellular membranes for forming ion channels 25. Therefore, it is possible that after silencing of CLIC1 gene expression, its ability in inserting into cellular membrane was attenuated, which led to a small number of cells that were able to penetrate through membrane in the CLIC1 siRNA group.

In summary, our study supported that CLIC1 gene silencing could promote apoptosis and inhibit proliferation of GBC cells. Owing to the rare malignancy of the GBC, the research of the effects of CLIC1 gene silencing on GBC cells is expected to be worthwhile in the treatment of this disease. And comprehensively considering the unique properties and functions of CLIC1 from the previous findings, the application of CLIC1 gene silencing may be possessed with feasibility to some extent. As this study did not provide thorough evidence on the potential mechanisms of CLIC1 gene silencing in promoting apoptosis and inhibiting proliferation of GBC cells, further large‐scale trails are needed to confirm this conclusion.

## Conflict of interests

None.
